The article "Arnica montana Stimulates Extracellular Matrix Gene Expression in a Macrophage Cell Line Differentiated to Wound-Healing Phenotype" was retracted in 2019. Reasons: a conflict of interest; concerns about the data; concerns about the results or conclusions.

# *Arnica montana* Stimulates Extracellular Matrix Gene Expression in a Macrophage Cell Line Differentiated to Wound-Healing Phenotype

**DOI:** 10.1371/journal.pone.0166340

**Published:** 2016-11-10

**Authors:** Marta Marzotto, Clara Bonafini, Debora Olioso, Anna Baruzzi, Laura Bettinetti, Francesca Di Leva, Elisabetta Galbiati, Paolo Bellavite

**Affiliations:** 1 Department of Medicine, University of Verona, Strada Le Grazie 8, 37134, Verona, Italy; 2 Department of Biotechnology, University of Verona, Strada Le Grazie 15, 37134, Verona, Italy; 3 Department of Biotechnology and Bioscience, University of Milano-Bicocca, Piazza della Scienza 3, 20126, Milano, Italy; University of Kansas Medical Center, UNITED STATES

## Abstract

*Arnica montana* (*Arnica m*.) is used for its purported anti-inflammatory and tissue healing actions after trauma, bruises, or tissue injuries, but its cellular and molecular mechanisms are largely unknown. This work tested *Arnica m*. effects on gene expression using an *in vitro* model of macrophages polarized towards a “wound-healing” phenotype. The monocyte-macrophage human THP-1 cell line was cultured and differentiated with phorbol-myristate acetate and Interleukin-4, then exposed for 24h to *Arnica m*. centesimal (c) dilutions 2c, 3c, 5c, 9c, 15c or Control. Total RNA was isolated and cDNA libraries were sequenced with a NextSeq500 sequencer. Genes with significantly positive (up-regulated) or negative (down-regulated) fold changes were defined as differentially expressed genes (DEGs). A total of 20 DEGs were identified in *Arnica m*. 2c treated cells. Of these, 7 genes were up-regulated and 13 were down-regulated. The most significantly up-regulated function concerned 4 genes with a conserved site of epidermal growth factor-like region (p<0.001) and three genes of proteinaceous extracellular matrix, including heparin sulphate proteoglycan 2 (HSPG2), fibrillin 2 (FBN2), and fibronectin (FN1) (p<0.01). Protein assay confirmed a statistically significant increase of fibronectin production (p<0.05). The down-regulated transcripts derived from mitochondrial genes coding for some components of electron transport chain. The same groups of genes were also regulated by increasing dilutions of *Arnica m*. (3c, 5c, 9c, 15c), although with a lower effect size. We further tested the healing potential of *Arnica m*. 2c in a scratch model of wound closure based on the motility of bone marrow-derived macrophages and found evidence of an accelerating effect on cell migration in this system. The results of this work, taken together, provide new insights into the action of *Arnica m*. in tissue healing and repair, and identify extracellular matrix regulation by macrophages as a therapeutic target.

## Introduction

*Arnica montana L*. (referred to here as *Arnica m*.) is one of the most popular medications in complementary medicine and is widely employed in tincture, ointment, cream, gel, and tablet form. It is a herb native to the mountains of Siberia and Central Europe, and has been used to treat various pathological conditions, including pain, stiffness and swelling associated with trauma, postoperative clinical conditions (including contusions and sprains) and for symptomatic relief in osteoarthritis [1–5]. As a herbal formulation, *Arnica m*. is generally applied only topically on the skin, while as a homeopathic formulation it is also given orally or as an injection—since it is not considered dangerous owing to the high dilution. The literature on *Arnica m*. in both phytotherapeutic and homeopathic preparations is rapidly increasing, but the knowledge of its action mechanism(s) remains scant.

The chemical composition of *Arnica m*. depends on the part of the plant that is used, principally the flowers and roots, and in general the most pharmacologically active compounds are sesquiterpene lactones, thymol derivatives, flavonoids, acid polysaccharides and their glycoconjugates [6–8]. The ability of *Arnica m*. to inhibit activation of transcription factors NF-κB and nuclear factor of activated T cells (NFAT) and pro-inflammatory cytokines IL-1 and TNF-α correlates with its quantitative and qualitative content of sesquiterpene lactones [9].

There is some experimental evidence, in laboratory animals, of an anti-inflammatory action of *Arnica m*. administered as crude ethanolic extract [10] or at the 6^th^ centesimal homeopathic dilution (6c) [11,12]. Additionally, *Arnica m*. treatment caused a reduction in inducible NO synthase and cyclooxygenase-2 protein levels, a reduction in TNF-α, and prevented nuclear translocation of NF-κB in J774 murine macrophage cells without cytotoxicity *in vitro* [13]. Furthermore, oral treatment with *Arnica m*. 30c protected experimental animals (rats) against hepatic mitochondrial membrane permeabilization induced by Ca^2+^ and lipid peroxidation due to the attack by reactive oxygen species [14].

Given the central role of macrophages in tissue repair and regeneration, we formulated the hypothesis that one of the cellular targets of *Arnica m*. action is the macrophage, and accordingly decided to evaluate this plant’s effects *in vitro* on the THP-1 human cell line, a widely used model for immune modulation [15,16]. This cell line is widely used in laboratories for the study of macrophage biochemistry and molecular biology. The advantage of a cell line resides essentially in the easier reproducibility of experiments in the same conditions, avoiding the variations due to individual sensitivity of different donors. Since we used very low doses of drugs—even with the highest *Arnica m*. 2c dilution, in assay medium the sesquiterpene lactones are in the 10^−8^ Mol/L dose—we expected small effect sizes and so preferred to use a highly reproducible model. THP-1 cells resemble primary monocytes, but when treated with low doses of phorbol esters (PMA) they differentiate to cells with the morphological and functional features of tissue macrophages. On the basis of environmental cues and molecular mediators, macrophages differentiate to either a pro-inflammatory type (M1) or to an anti-inflammatory or pro-reparatory type (M2) [17–20]. Accordingly, we used THP-1 macrophages polarized by interleukin-4 (IL-4) treatment to a phenotype that takes on characteristic properties functional to immune regulation, wound healing, and tissue remodelling [16,21].

In a preliminary study, we used RT-PCR analysis to investigate changes in the expression of a panel of 28 genes focused on immune response [22]. Among the tested genes, CXCL1 in particular exhibited the most substantial increase of expression, while CXCL2, CXCL8, BMP2 and NFKB1 were slightly up-regulated, suggesting a positive influence of *Arnica m*. on neutrophil recruitment and on angiogenesis. The most pronounced effects were noted in IL-4 polarized macrophages after 24h of *Arnica m*. treatment. Therefore, we decided to re-investigate the same cell extracts with the most high-throughput method, RNA-sequencing (RNA-seq), designed to evaluate the whole transcriptome. We assessed RNA samples from a series of 5 experiments testing *Arnica m*. at the 2nd centesimal homeopathic dilution (*Arnica m*. 2c) compared with vehicle (Control). This approach enabled us to identify all the potential genomic targets of the plant’s regulating action, through bioinformatics analysis of the differential expression of genes (*Arnica m*. 2c vs Control) and using statistical methods correcting for false discovery rate. Furthermore, since *Arnica m*. is used at several doses in clinical settings [5], we also tested pooled samples of the experiments carried out with higher dilutions, namely 3c, 5c, 9c and 15c. Lastly, to further investigate the potential therapeutic capacity of this plant, we tested *Arnica m*. and Control solutions using an *in vitro* model of wound healing, in which macrophages migrate through a scratch made in the culture cell monolayer. A major advantage of this method is that it mimics, to some extent, the migration of cells *in vivo* and is particularly suitable for studies on the effects of cell–matrix and cell–cell interactions during wound healing [23].

## Materials and Methods

### Materials

The human monocytic leukaemia cell line THP-1 was purchased from DSMZ (Germany). Growth media RPMI 1640, Ultraglutamine 20mM solution and DMEM with l-glutamine were purchased from Lonza (Belgium). Foetal bovine serum (FBS), phorbol 12-myristate 13-acetate (PMA), pure ethanol and ultra-pure water (W3500) were purchased from Sigma-Aldrich Co. (St. Louis, MO, USA). Human interleukin-4 (IL-4) was purchased from Macs-Miltenyi Biotec (Germany). Murine IL-4 was purchased from Peprotech (UK). Cell proliferation reagent WST-1 was purchased by Roche Diagnostics GmbH (Germany). RNeasy Mini kit was from Qiagen, (CA, USA). Ficoll-Hypaque and Percoll were purchased from GE Healthcare Life Science (Uppsala, Sweden).

### Test solutions

*Arnica m*. was produced by Boiron Laboratoires (Lyon, France) according to the French Homeopathic pharmacopoeia and provided as a first centesimal dilution (*Arnica m*. 1c) of the hydroalcoholic extract (Mother Tincture, MT) in 30% ethanol/distilled water. The content of sesquiterpene lactones of the MT was determined by liquid chromatography and the conformity of the whole extract to pharmacopoeia standards was checked by thin layer chromatography. UV-visible absorption spectrum of the *Arnica m*. 1c was performed with a Jasco V-650 double-beam spectrophotometer using quartz cuvettes with 1cm optical path and the vehicle ethanol 30% v/v as the reference-blank sample. Nanoparticle content was determined by nanoparticle tracking analysis (NTA) using the NanoSight LM10 (Malvern) instrument equipped with laser at 532nm and the NanoSight NTA 3.0 analysis software. Zeta potential was measured by Zetasizer Nano (Malvern) using disposable capillary cells (Malvern).

*Arnica m*. 1c was used to prepare the second centesimal dilution (*Arnica m*. 2c) by adding 50μl of 1c solution to 4.95ml of distilled ultra-pure water. Therefore, 2c corresponds to 10^−4^ of the MT. This solution was filtered with a 0.22μm Millipore filter and subjected to vigorous succussion with a Dyna-A mechanical shaker delivering 20 strokes/second with an 11mm travel distance. The Control test solution was prepared using 30% ethanol/distilled water (same batch of the *Arnica m*. 1c dilution) diluted 100x in distilled ultra-pure water and succussed as described for *Arnica m*. 2c sample. Final ethanol concentration in the cells was 0.03% v/v, since the test medicines were added as 10% of the final culture volume. This dose did not affect cell viability, as verified in preliminary experiments.

Higher dilutions of *Arnica m*. were prepared as described previously [22]. Starting from a 1c solution, serial 100x dilutions were prepared in 5ml of 30% ethanol/distilled water solvent followed by filtering and succussion. Stock *Arnica m*. dilutions in 30% ethanol/distilled water were wrapped in aluminium foil, stored at room temperature in the dark, and used within 12 months of preparation. The last centesimal dilution step was always performed immediately before each experiment, in ultra-pure water. Of the *Arnica m*. dilutions prepared in this way, those tested with the cells were: 2c, 3c, 5c, 9c, and 15c.

All procedures for drug preparation and cell treatments were done in sterile conditions.

### Cell cultures and treatments

The THP-1 cell line was cultured in RPMI 1640 medium, supplemented with FBS 10% and 2mM final concentration of Ultraglutamine (Lonza), at 37°C in 5% CO_2_ in a humidified incubator as described [22]. Briefly, in a typical experiment, on day one the cells were seeded at a density of 2.5x10^5^ cells/mL in 24-well plates in 1ml medium with 2mM Ultraglutamine and 2% FBS. On day 2 all the cell cultures were supplemented with 20 ng/mL of PMA and on day 3 the cultures were treated with IL-4 at a concentration of 50 ng/mL for 24h. On day 4 the plates were washed twice with culture medium and the cultures were again supplemented with 50 ng/mL IL-4 and incubated for 24h. Macrophages were exposed for 24h to *Arnica m*. dilutions or Control solvent (1ml cell culture + 110μl test solutions). We performed a total of 5 complete separate experiments; in each experiment, every treatment was performed in triplicate wells.

### Bone marrow–derived macrophages

For the scratch test, bone marrow–derived macrophages (BMDM) were isolated from femurs and tibias of 8 week-old wild-type C57BL/6J mice as described by Suen et al. (1999) [24] and Baruzzi et al. [25]. Briefly, cells were cultured in DMEM with Glutamax (Lonza) supplemented with 15% FBS, 10% L929-cell conditioned medium (LCM) as a source of colony-stimulating factor-1, 100 U/ml penicillin, and 100 μg/ml streptomycin (BMDM complete medium), and cultured at 37°C/5% CO2 in 75 cm2 flasks. After 24 h, the non-adherent cells were removed, counted, plated on bacteriological (non tissue-culture-treated) plastic dishes at a concentration of 1×10^5^/ml, and cultured in BMDM complete medium.

### Evaluation of cell viability

Cell viability was checked by the Cell proliferation reagent WST-1 assay. THP-1 cells were seeded at the density of 40000 cells/well in 96-well plates and differentiated with IL-4 as described above. After 24h of treatment with *Arnica m*. dilutions or with Control, 1:10 (v/v) pre-warmed WST-1 solution was added to the cells and the plate was incubated for 20 minutes. The absorbance (OD) of the samples was measured using a Victor3 multilabel reader (PerkinElmer, Shelton, CT, USA) at 450nm. Total proteins of cell extracts were quantified by Bradford assay according to the manufacturer’s instructions.

### RNA sequencing

Total RNA from cultured THP-1 cells was isolated using the RNeasy mini Kit (Qiagen). RNA quality and quantity were determined using a Nanodrop 2000 spectrophotometer (Thermo Scientific, Wilmington, DE). RNA samples were assessed for quality (integrity) using an RNA 6000 Nano Kit (Agilent, Wokingham, UK). The samples with RNA integrity numbers (RIN)>9 were considered adequate for library preparation. RNA aliquots (2.5μg) were used to isolate poly(A) mRNA for the preparation of a directional Illumina RNA-Seq library using the TruSeq RNA Sample Prep Kit v2 (Illumina Inc., San Diego, CA, USA). The quality of the library, before the generation of clusters, was checked with High Sensitivity DNA Kit (Agilent, Wokingham, UK) and the library was quantified by qPCR using the KAPA Library Quantification kit (Kapa Biosystems Inc., Woburn, MA, USA).

Libraries were sequenced with a NextSeq500 sequencer (HighOutput flow cell with 75 sequencing cycles) generating 75-bp sequences. The reads were aligned to the human reference genome (GRCh38) using the TopHat 2.0.14 software [26]. The expression value of known and novel genes was quantified as reads per kilobase of exon model per million mapped reads (RPKM) using the human working gene set (Ensembl release 80) as reference annotation. The effect of treatments was measured by calculating Log_2_ of the ratio between RPKM of each gene in *Arnica m*.-treated samples and Control-treated samples (Log_2_ Fold Change). Genes with Log_2_ Fold Change values that were significantly positive (up-regulated) or negative (down-regulated) were defined as differentially expressed genes (DEGs).

Sequences of DEGs in the “protein coding” category were functionally annotated using Blast2GO, assigning a GO term and a metabolic pathway in the Kyoto Encyclopedia of Genes and Genomes (KEGG) to the query sequences. Gene functional classification and enrichment analysis were performed by DAVID Bioinformatics Resources 6.7 (http://david.abcc.ncifcrf.gov) [27].The data discussed in this publication have been deposited in NCBI's Gene Expression Omnibus [28] and are accessible through GEO Series accession numbers GSE77381 and GSE77382 **(https://www.ncbi.nlm.nih.gov/geo/query/acc.cgi?acc=GSE77381; https://www.ncbi.nlm.nih.gov/geo/query/acc.cgi?acc=GSE77382).**

### Protein quantification by ELISA

Matrix-related proteins (fibronectin, fibrillin, and heparan sulfate proteoglycan 2) were quantified in conditioned medium of treated cells using ELISA assays fibronectin human Elisa kit (Abcam), human Fibrillin-2 ELISA Kit and human heparan sulfate proteoglycan 2 ELISA Kit (Cusabio), respectively.

### In vitro wound-healing (scratch) assay

The capacity of macrophages to close an artificial “wound” was assessed using a culture model in which a portion of a confluent BMDM monolayer was denuded of cells by scraping it with a pipette tip, after which the number of cells migrating into the open space was assessed microscopically [23]. Macrophages were cultured in 12-well plates in BMDM complete medium until confluent. On day 4, a portion of the cell cultures was supplemented with 20 ng/ml murine IL-4 while another portion was left untreated. On day 5 the monolayers were wounded by transversely scratching the well with the tip of a 200 μl pipette, tracing a 1 mm wide gap. The detached cells were carefully aspirated and the wells washed with phosphate-buffered saline (PBS). The medium during the migration test was DMEM (Glutamax, pen-strep) with 2% FBS, either with or without 20 ng/ml IL-4. *Arnica m*. 2c or Control solutions were added 24 h before wounding and maintained, during the migration time, at the concentration equal to 10% of the culture volume. Three sets of experiments were performed with triplicate wells for each condition. Photomicrographs of the central field of the wound were acquired by means of contrast phase microscopy using an Olympus IX50 microscope with 100x original magnification to assess cell migration. The experiments were evaluated by examining microscopically the cell migration front/border and using a grid composed of 500 small frames to calculate the % of wounded area occupied by macrophages.

### Statistics

RNA-seq analysis was performed separately on 5 experiments for *Arnica m*. 2c and Control solvent. For the analysis of RNA from cells treated with higher dilutions, RNA samples from 5 experiments carried out with *Arnica m*. 2c, 3c, 5c, 9c, 15c and Control solvent were pooled and sequenced.

The evaluation of differential gene expression between the *Arnica m*.-treated and Control samples from the RNA-seq data was performed using the DESeq2 package with a paired design [29]. Where indicated (Table 1), the p-values were corrected for the False Discovery Rate (FDR) with the Benjamini and Hochberg method using an adjusted p-value threshold of 0.05 [30]. Comparisons were done by testing, for each gene and each experiment (N = 5), the null hypothesis that the Log_2_ Fold Change was exactly zero, i.e., that the gene was not at all affected by the treatment.

**Table 1:** Gene expression of IL-4 differentiated THP-1 macrophages, treated with Control solvent or *Arnica m*. 2c (n = 5).

Effect	HGC Nomenclature		RPKMIL-4 Control		RPKMIL-4 + *Arnica m*.		Log_2_ Fold Change			Description
	Symbol	ID	Mean	SE	Mean	SE	Mean	SE	P value(corrected for FDR)	
Up-regulated	CR1	2334	1.6	0.4	2.0	0.5	**0.3**	0.07	0.0225	Complement component (3b/4b) receptor 1
	LRP1	6692	19.4	2.0	23.6	2.0	**0.29**	0.05	< 0.0001	Low density lipoprotein receptor-related protein 1
	FN1	3778	426.3	30.8	509.5	23.4	**0.27**	0.05	0.0007	Fibronectin 1
	FBN2	3604	3.0	0.2	3.6	0.1	**0.27**	0.09	0.0418	Fibrillin 2
	HSPG2	5273	9.5	1.3	11.3	1.5	**0.25**	0.09	0.0332	Heparan sulfate proteoglycan 2
	KMT2D	7133	6.3	0.4	7.5	0.3	**0.24**	0.06	0.0037	Lysine (K)-specific methyltransferase 2D
	MACF1	13664	2.5	0.1	2.9	0.1	**0.24**	0.08	0.0379	Microtubule-actin crosslinking factor 1
Down-regulated	COX3	7422	529.6	23.7	448.8	18.0	**-0.24**	0.05	0.0418	Mitochondrially encoded cytochrome c oxidase III
	ND2	7456	4766.7	289.3	3982.6	184.5	**-0.25**	0.04	0.0038	Mitochondrially encoded NADH dehydrogenase 2
	COX1	7419	1798.3	60.5	1506.3	46.7	**-0.25**	0.07	0.0418	Mitochondrially encoded cytochrome c oxidase I
	ND6	7462	85.2	4.4	70.2	1.8	**-0.27**	0.04	0.0018	Mitochondrially encoded NADH dehydrogenase 6
	ATP6	7414	404.9	15.1	334.1	11.3	**-0.28**	0.04	0.0008	Mitochondrially encoded ATP synthase 6
	ND5	7461	392.7	24.5	321.2	8.1	**-0.28**	0.06	0.002	Mitochondrially encoded NADH dehydrogenase 5
	ND1	7455	2081.5	112.5	1690.4	68.2	**-0.3**	0.061	0.0008	Mitochondrially encoded NADH dehydrogenase 1
	ND4	7459	819.0	41.2	659.1	16.6	**-0.31**	0.06	0.0006	Mitochondrially encoded NADH dehydrogenase 4
	MTRNR2L8	37165	45.6	4.1	36.3	1.4	**-0.31**	0.088	0.0176	MT-RNR2-like 8
	CYTB	7427	35.1	2.2	28.1	1.5	**-0.32**	0.057	0.0001	Mitochondrially encoded cytochrome b
	CCDC88B	26757	5.4	0.5	4.3	0.3	**-0.32**	0.068	0.0078	Coiled-coil domain containing 88B
	ATP8	7415	1530.0	85.2	1218.2	38.6	**-0.32**	0.094	0.0135	Mitochondrially encoded ATP synthase 8
	ND4L	7460	102.6	7.4	79.5	2.0	**-0.36**	0.088	0.0006	Mitochondrially encoded NADH dehydrogenase 4L

The statistical significance of the differences between expression profiles of gene groups (Up-regulated and Down-regulated genesets) from cells treated with various *Arnica m*. dilutions (2c, 3c, 5c, 9c, 15c) was calculated by the Friedman multi-sample test followed by the Wilcoxon signed-rank test using the SPSS software, version 17 (SPSS Inc., Chicago, IL, USA). The Friedman test is a nonparametric test for multiple related samples (in this case, the multiple genes– 7 up-regulated or 13 down-regulated—from cells treated with five *Arnica m*. dilutions and control solution) that checks the null hypothesis that multiple ordinal responses in terms of RPKM come from the same population. After verifying the significance of the Friedman test, we used the Wilcoxon signed-rank test for paired data to evaluate the differences between RPKM of genes after treatments with each *Arnica m*. dilution and mean RPKM of Control-treated cells, and to check whether such differences were prevalently positive or negative, or evenly distributed between the two signs. The differences were accordingly ranked, and the positive and negative ranks were separately summed and statistically compared using the specific Wilcoxon tables. The logic of this approach is to test the null hypothesis of the absence of treatment effects: if treatment has no effect the differences between gene expression (RPKM) of *Arnica m*.-treated samples and Control-treated samples should approach zero in all considered genes of the group. Moreover, since some gene may be modified by chance, the number of up- and down- regulated genes should be approximately the same in a given group (not significantly different). Log_2_ Fold Changes were lower than or equal to ±0.05 (-0.05<FC<0.05) were considered to be null.

Comparison of protein release in *Arnica m*. 2c and Control samples was done with the Sigma Plot statistical package using the paired t-test, or the Wilcoxon Signed Rank Test when data were not normally distributed (as preliminarily evaluated by Shapiro-Wilk normality test). Cell viability data were evaluated by ANOVA followed by Dunnet post-hoc test, using the SPSS statistical package.

Statistical evaluation of the scratch assay was done using the Friedman test. It is used to test for differences between groups (in this case the series of time points for the Treated and Control samples) when the dependent variable being measured is ordinal. The null hypothesis is that the time series for two compared treatments (*Arnica m*. and Control solvent) will be equal.

## Results

### Characterization of *Arnica m*.

The *Arnica m*. 1c used the starting material for this series of experiments was analysed by physicochemical approaches. Fig 1 shows the UV-VIS absorption spectrum. This was characterized by a large UV peak around 220 nm, followed by two shoulders at 280nm and 340nm. No substances absorbing at wavelength > 500 nm were detected in our preparation.

**Fig 1:** Absorption spectrum of *Arnica m*. 1c used as starting material.

NTA analysis of the original *Arnica m*. 1c sample revealed the presence of a heterogeneous and polydisperse quantity of nanoparticles (9.3 ± 1.0 particles/frame) corresponding to a concentration of 1.83 x 10^8^ ± 1.88 x 10^7^ particles/ml. The NTA spectrum (Fig 2) showed a profile with about 6 peaks with a hydrodynamic diameter ranging from 100 to 500nm and a mean size of 274.4 ± 100.4 nm. Zeta potential of these nanoparticles was -25.54 ± 9.50 mV (n = 12 determinations).

**Fig 2:** Nanoparticle spectrum of *Arnica m*. 1c. used as starting material. The line is the average of 10 replicate measurements and vertical bars indicate SD.

The amount of total sesquiterpene lactones in the original Mother Tincture was 36 mg/100ml. Since the mean molecular weight of *Arnica m*. sesquiterpene lactones is 340 g/mol [31], this amount is equivalent to 1.05 x 10^−3^ Mol/L and the calculated concentration of these active substances is 1.05 x 10^−5^ Mol/L in *Arnica m*. 1c and 1.05 x 10^−7^ Mol/L in *Arnica m*. 2c (final concentration in assay = 1.05 x 10^−8^ Mol/L).

### Cell viability

The WST assay of cell viability (Fig 3) showed that the metabolic activity of macrophages, both in the resting state and after IL-4 differentiation, was slightly increased after 24h incubation with *Arnica m*. dilutions 2c and 3c, but the difference with the Control vehicle was not statistically significant. Since the WST-1 assay depends on the level of NADH produced by the cells [32], this result shows that mitochondrial NADH-producing activity was not significantly impaired by *Arnica m*. Interestingly, WST reduction was higher in IL-4 differentiated macrophages, irrespective of the presence of *Arnica m*., suggesting that this cytokine stimulates the basal metabolism of macrophages.

**Fig 3:** Cell viability of macrophages. THP-1 macrophages in the resting state (diagonal bars) or after differentiation with IL-4 (crossed bars) were cultivated for 24 hours in the presence of *Arnica m*. at various dilutions or Control solvent. The histograms report mean values ± SE of 6 separate wells of a typical experiment. There are no significant differences between any *Arnica m*. dilution and Control (p>0.05)

### Changes in gene expression after *Arnica m*. treatment

The effects of *Arnica m*. treatment on the global gene expression of IL4-polarized THP-1 cells were investigated after 24h of incubation by comparison with Control. The basic RNA-seq analysis were done in cells treated with *Arnica m*. 2c –the lowest dilution and highest dose that could be used since 1c contained a dose of ethanol incompatible with cell culture—and were reproduced in 5 different biological replications. Approximately 25 million valid reads obtained for each sample sequencing were unambiguously annotated on 60434 gene transcripts. No arbitrary filtering of expression level was applied to the dataset. Differential gene expression analysis was performed to identify significant target genes of *Arnica m*. 2c action. A list of 20 statistically significant DEGs was thus obtained as shown in Table 1. The RPKM and Log_2_ Fold Changes values of all the 5 separate experiments performed, plus the original values of pooled samples from assays done with higher dilutions, are reported in S1 Table.

Mean RPKM is an indicator of the absolute amount of RNA in samples from cells treated with *Arnica m*. or Control solution. Table 1 shows that FN1 (fibronectin) was by far the most expressed gene and its RPKM values increased from 426.3 to 509.5. The second most expressed gene was LRP1 (from 19.4 to 23.6), and the third was HSPG2 (from 9.5 to 11.3). The down-regulated genes included 6 mitochondrially-coded NADH dehydrogenases which are subunits of Complex I, Cytochrome B of Complex III, 2 Cytochrome oxidases of Complex 4, and two ATP synthases of Complex V. In eukaryotes, the hydrophobic core subunits of Complex I are encoded by the mitochondrial genome [33] and are normally highly expressed. We confirmed this high gene expression in Control (e.g. 529.6 RPKM for cytochrome c oxidase III, 4766.7 RPKM for NADH dehydrogenase) and *Arnica m*. caused a slight but reproducible decrease of the expression of all the indicated genes (Table 1 and S1 Table).

Mean fold changes, calculated as the average of the Log_2_ Fold Change of the 5 replicates, ranged from 0.30 (maximum up-regulation) to -0.36 (maximum down-regulation). The 7 up-regulated genes included low-density lipoprotein-receptor-related protein 1 (LRP1), fibronectin 1 (FN1), lysine (K)-specific methyltransferase (KMT2D), complement component receptor 1 (CR1), heparan sulfate proteoglycan (perlecan, HSPG2), microtubule-actin crosslinking factor 1(MACF1), and fibrillin 2 (FBN2). The set of down-regulated DEGs (13 genes) were mitochondrial genes coding for proteins of the mitochondrial respiratory chain complex.

Functional gene enrichment analysis (Table 2) was performed by analysing international databases of gene sequences using the DAVID software. Among the genes stimulated by *Arnica m*, a statistically significant enrichment of genes with EGF-like (LRP1, HSPG2, FBN2, FN1) and Calcium ion binding motifs (LRP1, MACF1, FBN2) emerged (Fisher p<0.001 and <0.05 respectively). Most notably, a clearly up-regulated function concerned the proteinaceous extracellular matrix (ECM), including genes HSPG2, FBN2, FN1 (p<0.01). The down-regulated genes converge into the common pathway of oxidative phosphorylation and particularly into the cell component gene ontology of mitochondrial complex I as expected (p<0.001).

**Table 2:** Functional classification and gene enrichment analysis.

Geneset	Database	Function ID	Description	Fold Enrichment	P value	Genes
Up-regulated	INTERPRO	IPR013032	EGF-like region, conserved site	**32.49**	**<0.001**	LRP1, HSPG2, FBN2, FN1
	GOTERM_CC	GO:0005578	Proteinaceous extracellular matrix	**17.12**	**<0.01**	HSPG2, FBN2, FN1
	GOTERM_MF	GO:0005509	Calcium ion binding	**7.06**	**<0.05**	LRP1, MACF1, FBN2
Down-regulated	GOTERM_CC_FAT	GO:0005747	Mitochondrial respiratory chain complex I	**101.44**	**<0.001**	ND1, ND4L, ND4, ND5, ND2, ND6
	KEGG_PATHWAY	hsa00190	Oxidative phosphorylation	**26.08**	**<0.001**	ND1, ND4L, ND4, COX3, ND5, COX1, ND2, CYTB, ATP8, ND6, ATP6

### Protein release in supernatants

To confirm the function of up-regulated genes, we measured the release of some relevant proteins of ECM in cell supernatants. Of these, HSPG2 and fibrillin were detected only in traces, while fibronectin was identified in considerable amounts (Table 3). This protein was increased in IL-4 macrophages as compared with non-polarized cells and was increased by *Arnica m*. 2c treatment.

**Table 3:** Proteins detected in supernatant of THP-1 macrophages cultivated 24 h in the presence and absence of *Arnica m*. 2c.

		Normal Macrophages			IL-4-polarized Macrophages		
		*Arnica m*. 2c	Control	p	*Arnica m*. 2c	Control	p
HSPG2(Perlecan)	Mean	0.43	0.42	n.s.	0.35	0.31	n.s.
	SD	0.12	0.18		0.09	263	
Fibrillin	Mean	0.002	0.005	0.065	0.0004	0.0004	n.s.
	SD	0.001	0.0003		0.0004	0.0004	
Fibronectin	Mean	1.62	1.41	0.063	22.91	17.49	0.031
	SD	0.65	0.51		22.21	15.50	

PMA-differentiated THP-1 macrophages were polarized with IL-4 as described in Methods or maintained in the same medium without IL-4 (Normal Macrophages), then both cultures were incubated for 24 h in the absence (Control) or in the presence of *Arnica m*. 2c. N = 6 complete experiments, assay in technical duplicates (HSPG2 and fibrillin) or triplicates (fibronectin). Values are micrograms/million cells. Note that HSPG2 and fibrillin in some experiments were under the detection limit of the assays.

Fig 4 shows the amount of fibronectin detected in the supernatants in the 6 separate experiments. In IL-4 macrophages, the *Arnica m*. 2c effect was almost null in one experiment only, while in the other 5 it ranged from 13.9% to 39.6% (p<0.05).

**Fig 4:** Fibronectin detected in supernatants of cell cultures in the absence and in the presence of *Arnica m*. 2c. Symbols indicate the fibronectin values of the same experiments in the two conditions of polarization. The reported values are percent effect as compared with Control of the same experiment.

### Testing higher *Arnica m*. dilutions

We then investigated the changes induced by increasingly higher *Arnica m*. dilutions in the same genes that had shown statistically significant alterations after treatment with 2c test solution (Table 1). These effects are reported in Fig 5 as Log_2_ Fold Changes in comparison with the mean of Controls and the RPKM of all samples are given in S1 Table, right part. Owing to technical constraints (availability of sufficient volumes) and the high costs of RNA-seq, we could not separately assay gene expression changes for all five experiments at all the various dilutions. Therefore, to decrease experimental variability, we pooled RNA from samples of cells treated with the same *Arnica m*. dilution, using extracts from all the five experiments performed. This approach reduced the variation possibly due to biological replicates, but meant we could not evaluate the standard errors of each separate gene. For these reasons, Fig 5 (panels B-F) does not include the error bars for individual genes, but only a mean value and standard error for each group of genes (7 up-regulated in red, 13 down-regulated in blue). Since most of genes in up- and down-regulated genesets belong to similar functional groups, calculating the mean of the various genes provided a first and preliminary evaluation of the major effects across different dilutions.

**Fig 5:** Effects induced by increasing dilutions of *Arnica m*. on gene expression in THP-1 cells. DEGs described in Table 1 were divided in the two groups as upregulated (red bars) and down-regulated (blue bars) genesets. Grey bars report the mean fold changes ± SE of the two genesets at each dilution tested. Panel A: *Arnica m*. 2c Log_2_ fold change values calculated from 5 experiments; Panels B-F *Arnica m*. 2c, 3c, 5c, 9c, 15c Log_2_ fold changes values of pooled RNAs of 5 experiments. P values of Wilcoxon signed-rank test statistics are reported near the mean of each geneset.

The gray bars in Fig 5 show the means and standard errors of the *Arnica m*. effects for each geneset (up-regulated and down-regulated), with the p values of the differences between treatments and Control solvent. By Wilcoxon statistics we can test the null hypothesis that treatment has no effect: in such a case the mean fold change values for a given group of genes should approximate zero, and eventually (since some genes may be modified by chance), the mean of all considered genes should approach zero. Finally, if the null hypothesis is true, the number of up- and down- regulated genes–assuming random up-regulation or down-regulation—should be approximately the same.

Considering the *Arnica m*. 2c dilution (Fig 5, top two panels) we can see that the up-regulated and down-regulated groups of genes responded in the pooled analysis (Panel B) roughly in the same direction as they did in the separate analysis (Panel A). More generally, looking at the red bars (which denote the genes previously found to be up-regulated) we see that, among these, 7 out of 7 were also up-regulated in this pooled analysis. Conversely, looking at the blue bars (denoting genes previously found to be down-regulated) we see that all 13 of these genes are likewise down-regulated in this pooled analysis. This indicates that the values of pooled samples were reliable also if done with a single RNA-seq assay. The differences with the Control were evaluated statistically only for each entire geneset (up-regulated or down-regulated groups of genes) by applying the Wilcoxon signed-rank test for paired data, testing whether the differences are mainly positive or negative, or evenly distributed between the two signs. The changes due to *Arnica m*. 2c were highly significant both in the mean of 5 experiments (Panel A) and in the pooled samples (Panel B). Absolute fold changes less than or equal to 0.05 were considered null.

For what concerns the higher dilutions, *Arnica m*. 3c (Panel C) similarly showed a prevailing stimulating effect in the previously up-regulated geneset: 6 genes out of a total of 7 (the exception was MACF1) were here also be found up-regulated, while 12/13 genes of the previously down-regulated geneset were actually down-regulated also here (the exception was CCDC88B). The global changes of each geneset (grey bars) were approximately of the same magnitude as those induced by *Arnica m*. 2c and were statistically significant. *Arnica m*. 5c (Panel D) instead stimulated all genes of the up-regulated geneset in a statistically significant way and the prevailing inhibiting effect was also confirmed on the down-regulated geneset, with the exception of ATP8 which was unchanged and of CCDC88B that showed an inversion of effect. *Arnica m*. 9c has a very faint effects in either direction, that was variable in different genes, so that the global analysis was at limit of statistical significance threshold for the up-regulated geneset. On the downregulated geneset *Arnica m*. 9c had a faint but statistically significant effect, with the exceptions of ATP8 and CCDC88B. *Arnica m*. 15c slightly up-regulated 7 genes out of a total of 7, the strongest effect was on HSPG2. Considering the downregulated geneset, *Arnica m*. caused a slight but consistent downregulation of 10 genes, had no effect on 2 (ND6 and ATP8) and upregulated CCDC88B as seen with the lower dilutions. In summary, both upregulating and downregulating effects were maintained across the increasing dilutions, while for many considered genes a non-linear trend in the dose-responses appeared.

### Other candidate DEGs

The results presented thus far concern significant alterations of a series of genes identified through the transcriptome screening and analysis under very stringent statistical tests—that is, after adjusting for FDR. By so doing, we decrease the probability of type-1errors but also the probability of discovering true positive effects of *Arnica m*. on other candidate genes that are involved in ECM. In point of fact, a large list of proteins with different roles are involved in the ECM changes that occur during the various phases of wound healing and remodeling and includes various cell types. To explore the possible involvement of other candidate genes in the *Arnica m*. effects on macrophages, we performed a further analysis which included all the DEGs with a p value < 0.05 without applying the correction (n = 476). We then searched for the list of proteins interacting with fibronectin in the Reactome database (http://www.reactome.org/) and retrieved a list of 291 genes that represent the pathway of extracellular matrix organization (identifier R-HSA-1474244.1). By matching these 291 genes with the 476 differentially expressed upon *Arnica m*. 2c treatment, we retrieved 22 genes, 13 of which were upregulated and 9 downregulated. The upregulated genes included FN1, FBN2 and HSPG2 as expected, plus fibrillin 1, nidogen, osteonectin, dystonin, MMP2 and ADAMTS2. Two collagen genes, two metallopeptidases and the proteolytic enzyme calpain 3 resulted among the down-regulated DEGs. The new genes (apart those already discovered with application of FDR and cited in Table 1) are reported in S2 Table, left part. The expression of other important proteins—e.g. periostin, osteopontin or tissue inhibitor metallopeptidases–does not appear to be affected.

We also checked whether the same genes were affected by increasing drug dilutions (S2 Table, right part), but results were much less regular than those observed with the group of genes described in Table 1 and Fig 5. Even if a general tendency to respond in the same direction could be noted, most genes changed from up to down regulation or did not change with an inconsistent way. Only the genes ADAMTS2 and ITGAD responded to *Arnica m*. treatment in the same way (upregulation and down-regulation respectively) in cells treated by all dilutions. Although this supplemental analysis should be considered only as preliminary indication of further genes involved, it suggests that in *Arnica m*. may affect ECM organization in a broad and complex way.

In a previous study, which analysed a panel of inflammatory genes by RT-array, *Arnica m*. stimulated the expression of BMP2, CCL2 (MCP-1), CXCL1, CXCL2, CXCL8, MRC1, NFKB1 and inhibited the expression of MMP1 and TNFA [22]. The present analysis, carried out on whole transcriptome with RNA-seq, confirmed the same trend of expression changes in the majority of those genes, albeit with values that do not attain statistical significance (data not shown). Of the previously described genes, the only ones whose trend was not confirmed by RNA-seq were NFKB1 and TNFA, which did not change upon *Arnica m*. treatment according to the present RNA-seq analysis. It should be noted that RNA-seq is a high-throughput technique with higher dynamic range compared to gene-focused RT-PCR, a factor that may explain a partial discrepancy between the two methods, particularly in case the interested genes have low expression values.

### Effectiveness on a wound healing model

In order to investigate the possible functional implications of the observed molecular changes, a migration test was performed on cells treated with *Arnica m*. 2c comparing them with untreated cells. The scratch assay is an easy, low-cost and well-established method for measuring cell migration *in vitro* [23]. The test is based on the observation that, when a new artificial gap–referred to as “scratch”–is created on a confluent cell monolayer, the cells on the edge of the newly created gap will move into the opening to close the gap. To test *Arnica m*. in this system we used primary mouse bone marrow derived macrophages rather that THP-1 cells. This because in the previous experience of our department laboratory, and in our own test assays, the mouse cells formed more stable monolayers and showed more consistent motility [25]. The left panels of Fig 6 show some typical features of the scratch test assay.

**Fig 6:** Wound closure effect of *Arnica m*. Light microscope images of *in vitro* wound closure using a confluent monolayer of BMD macrophages. The microphotographs show one representative experiment of cell migration into the created wound area in the absence (A and C) and in the presence (B and D) of *Arnica m*. 2c. Images A and B show the wound area immediately after scratching, while C and D show the wound area after 4.5 h. Pictures were acquired by means of contrast phase microscopy with 100x original magnification. The bar charts (E and F) report the gap width of the wound area before and after cell migration. E and F: Time-course of wound occupancy in the absence (E) and in the presence (F) of 20 ng/ml IL-4. Gray bars: Control solvent, yellow bars: *Arnica m*. 2c. Means±SE of three replicate wells of an experiment representative of the three performed. The result of the Friedman test comparing the whole series of changes in cells treated with drug or with Control solvent is reported in the graph panels.

Standardized scratches initially caused complete removal of the monolayers of BMD macrophages (Fig 6A and 6B). However, after a few hours the cells started to fill the gap sufficiently to allow the front line to be easily determined and the covered surface quantified. In the presence of *Arnica m*. (Fig 6D) the filling of the gap was slightly faster than in its absence (Fig 6C), particularly in the presence of IL-4. The same field was completely full of macrophages after 24 hours of incubation in the presence of IL-4 (98.8±0.7% occupancy with Control cells and 99.3± 0.1% with *Arnica m*., treated cells, n.s.) while in the absence of IL-4 a smaller part of the gap was filled (63.2±3.9% occupancy with Control cells and 62.3±7.0% with *Arnica m*. treated cells, n.s.) (data not shown in figure). The bar charts on the right of Fig 6 represent the time-course of cell migration in the absence (E) and presence (F) of IL-4. *Arnica m*. 2c promoted a faster cell migration in both conditions but the difference between drug and Control was higher and statistically significant only in the presence of IL-4 (p = 0.014). The level of wound closure with the remedy was about 30% higher than that obtained with the Control solvent.

## Discussion

Preparations from traditional medicinal plants are often used as alternative remedies aimed at facilitating wound healing and tissue repair [34,35]. However, according to the available literature in medical databases, the mechanisms of the wound-healing effects of homeopathic remedies have yet to be fully understood. The application of whole plant extracts, at suitable dilutions and formulations, may be beneficial because herbaceuticals can have multiple and pleiotropic targets [36]. *Arnica m*. is widely used to treat various pathological conditions such as bruises, swelling associated with trauma, pain, inflammation, wounds and post-operative clinical conditions [3,5,37,38]. Investigations of its cellular and molecular targets have focused on inflammatory pathways, but little is known about its possible action on the stages of tissue formation and renovation. To fill this gap, we evaluated different dilutions of the whole plant extract in THP-1 human cells, differentiated into an IL-4 activated phenotype involved in wound healing and tissue remodelling. RNA sequencing of whole transcriptome allowed the identification of several genes whose expression was significantly altered following the treatment.

The physicochemical features of the *Arnica m*. used as a starting material to prepare further working dilutions were investigated through NTA, which provided a quantitative and morphological analysis of nanostructures in the solution. Nanostructures can form naturally during preparation of herbal extracts in liquid solution, and the presence of traces of silica from the glass container has been observed to help nanoparticle nucleation [39]. Moreover, exosomes or lipidic plant debris may be present in plant extracts [40]. In this work, for the first time, *Arnica m*. preparations were found to exhibit polydispersed nanostructures, ranging from 100 to 400 nm in size. These nanosized formations might represent a bioactive form of diluted herbal extracts, as some authors have suggested [41–44], and this interesting hypothesis deserves further investigation.

The main and novel finding was the increased expression of several genes of tissue matrix proteins and particularly of fibronectin, whose increase was confirmed also by protein assay in culture supernatants. This evidence suggests a new and relevant property of this plant in wound-healing processes. In fact, most of the up-regulated genes which emerged from this study belong to the extracellular matrix (ECM), and their enrichment as a functional group of genes is highly significant. The ECM is composed of collagens, proteoglycans/glycosaminoglycans, elastin, fibronectin, laminins, fibrillin, and several other glycoproteins. Matrix components bind to each other as well as to cell adhesion receptors, forming a complex network by which cells reside in connective tissue and epithelial cells bind to basement membrane and fibrillar components.

Fibronectin is a multi-domain protein with an essential role in the ECM since it binds to both cell receptors and connective tissue fibres. Cell receptors for fibronectin transduce signals which regulate diverse functions, such as survival, growth, and migration, whose regulation is vital during normal and pathological conditions [45,46]. This protein is vital for establishing and maintaining three-dimensional tissue architecture and for regulating cellular processes including adhesion, spreading, proliferation, and migration [47]. Fibronectin supports efficient platelet aggregation and pro-coagulant activity [48]; in the wound site it is also vital for regulating the neovascularisation of granulation tissue during the resolution of tissue injury. Fibronectin production appears to be an important component of the early tendon repair process [49,50]. FN-1 gene is overexpressed in macrophages during the healing phase of inflammation, suggesting it has important role in ECM deposition and tissue remodeling in acute inflammatory reactions and in chronic inflammatory diseases [51]. Based on these considerations, we can formulate the hypothesis that even a modest increase (20–30%) in the production of fibronectin induced by treatment with *Arnica m*. could greatly facilitate the consolidation of the wound and the migration of epithelial cells over the granulation tissue.

Other up-regulated genes included LRP1, HSPG2, and FBN2, which have an EGF-like domain in common with FN1. The highly significant association of these four genes into this functional group defined by enrichment analysis strengthens the conclusion that the described changes of gene expression identify specific *Arnica m*. targets and can not be a result of chance. EGF-like domain is an evolutionary conserved domain, which derives its name from the epidermal growth factor, which has an important role in cell growth and tissue repair. Most occurrences of the EGF-like domain are found in the extracellular domain of membrane-bound proteins or in proteins known to be secreted, such as components of the extracellular matrix. The presence of the EGF-like domain is important in protein-protein interactions and the proteolytic release of this domain from membranes may have paracrine activity on erbB receptors involved in cell growth and survival [52]. The interaction between the EGF-like domain and other ligands is often calcium-dependent, a feature that is in keeping with the enrichment of calcium-binding group of genes.

Low-density lipoprotein-receptor-related protein-1 (LRP1) is a receptor that mediates endocytosis and is coupled to activation of cell signaling. LRP-1 binds and internalizes numerous, structurally diverse ligands, delivering most but not all these ligands to lysosomes for degradation [53]. LRP-1 also controls the plasma membrane proteome by regulating maturation and transport of proteins in the secretory pathway [54]. Recently, its role as a regulator of inflammation has emerged, probably linked to its capacity to bind extracellular matrix proteins including fibronectin and thrombospondin [55] and to clear metalloproteinases [56]. The ability of macrophage LRP1 to modulate endocytosis and protein degradation confers on it a role in restoring connective tissue integrity after wound and inflammation—eg. adhesion and deadhesion processes, cell movements, clearance of growth factors and proteases (e.g. MMP) that are generated in an inflammatory environment. In addition, LRP1 regulates matrix deposition, in part, by modulating levels of connective tissue growth factor [57]. Finally, LRP-1 affects macrophage polarization and promotes the development of an anti-inflammatory M2 functional phenotype [58].

Heparan sulfate proteoglycan 2 (HSPG2, Perlecan) is a protein that in humans is encoded by the HSPG2 gene, present as a core protein in basement membrane. HSPG2 is a key component of the cortical bone and serves as a tethering element that connects the osteocyte cell body to the bone matrix. A reduction in perlecan secretion interferes with bone response to mechanical loading in vivo [59].

The protein encoded by KMT2D is a histone methyltransferase that methylates the Lys-4 position of histone H3, an event which regulates chromatin accessibility of adjacent genes and is associated with positive regulation of transcription. The epigenetic modifications induced by this protein, which are slight even after *Arnica m*. 2c treatment, may have a biological role that remains to be identified. In fact, many genes are expressed under the presence of this histone modification, e.g. the genes considered markers for M2 phenotype in IL-4 treated macrophages [60]. The gene MACF1 (microtubule and actin crosslinking factor 1) is likewise slightly but significantly overexpressed by *Arnica m*. 2c treatment. This protein has the ability to bind directly to and crosslink microtubules and F-actin networks, thereby directing microtubule organization. Directional cell movement is essential for wound repair, and MACF1 has been observed to play a role in wound healing and epidermal migration. MACF1 activity is in fact required for rapid and efficient formation of a hyperproliferative epithelium in response to injury, and its function is exerted primarily on epidermal migration rather than proliferation [61].

The decreased expression of several mitochondrially-coded genes of respiratory chain is a puzzling result. Assuming that this phenomenon was accompanied by a decreased synthesis of related proteins, one would envisage a decreased rate of respiratory chain and oxidative phosphorylation. Certainly, this expression change was not associated with lack of metabolic energy or toxic damage, since cell viability was not changed upon *Arnica m*. treatment. Instead, the slight increase of WST-1 reduction (not statistically significant, and to be confirmed by further studies) could suggest an increased level of intracellular NADH [32] as a consequence of decreased consumption in the mitochondrial respiratory chain. Furthermore, since the mitochondrion is a source of free radicals in conditions of lack of oxygen and reperfusion [62], it is possible that a moderate decrease of respiratory chain rate could have a cytoprotective effect in conditions of lack of oxygen, such as those presumably encountered by the cells in wounded tissue. This hypothesis is in agreement with the finding that a 30c dilution of *Arnica m*., administered orally to laboratory rats, decreased oxygen consumption of isolated liver mitochondria and protected from oxidative damage caused by lipid peroxidation [14]. The authors of that work interpreted this effect as a defence against oxidative stress. Furthermore, in fibroblast-like cells, whole extract of *Arnica m*. showed antioxidant activity and a cytoprotective effect against oxidative damage [63]. Only one paper reports an inhibitory action of *Arnica m*. on nitric oxide and TNF-α production by murine macrophages [13]. In our model of *in vitro* wound, treatment with *Arnica m*. 2c increased cell motility, confirming that the drug does not influence in a negative way the energy metabolism of the cell.

Among the down-regulated genes, the only non-mitochondrial gene was CCDC88B, coding for coiled-coil domain containing protein 88b, that is expressed in lymphocytes and myeloid cells and may have a role in regulation of T-cell function during inflammation [64]. Interestingly, this gene showed an unusual behaviour in cells treated with different dilutions (Fig 5): its expression decreased in samples from cells treated with low dilutions of *Arnica m*. (2c and 3c) while it increased in those treated with higher dilutions.

One of the major components of *Arnica m*. with an acknowledged biological activity is the sesquiterpene lactone helenalin, known for its anti-inflammatory properties. In a lymphoid cellular model, helenalin was found to inhibit the transcription factor NF-kappaB—a central mediator of human immune response—through the alkylation of p65 subunit (RelA), thus preventing its binding to DNA [6]. However the cited studies did not evaluate the contribution of the whole plant extract and used helenalin at a concentration of 10^−5^ Mol/L, much higher than that present in *Arnica m*. 2c used in this investigation, which had a final concentration in assay of 1.05 x 10^−8^ Mol/L. In this RNA-seq investigation, NFKB1 and RELA gene expression were not modified by *Arnica m* but, the reported effects of helenalin on NF-kappaB were due the inhibition of protein activation, rather than to an effect at the transcription level. The role of the NF-kb system and other transduction factors in the regulation of fibronectin synthesis and in the effects of *Arnica m*. remains to be further investigated.

Our findings provide a firm molecular explanation for previous experimental observations reporting significant effects of *Arnica m*. on inflammation and wound healing processes. In a randomized double-blind study conducted on humans, *Arnica m*. at a low homeopathic dilution (4x) reduced wound irritation (redness, swelling and heat) after hallux valgus surgery and ameliorated postoperative conditions in fewer days than did diclofenac [37]. An anti-inflammatory effect of *Arnica m*. (6c dilution) on carrageenan-induced foot oedema in rats has been reported by some authors [12] and a complex homeopathic product based on *Arnica m*. plus other compounds at low dilutions (4x-6x) was effective for blood-induced experimental oedema [65,66]. *Arnica m*. 3x as a topical gel improved the healing of surgically-induced wounds in Wister rats, but significant differences were noted only when the drug was delivered together with microcurrent application [67]. A commercial homeopathic complex containing a low dilution (4^th^ decimal, 4x) of *Arnica m*., *Calendula* and *Hypericum* promoted fibroblast growth in a scratch model of cellular wound closure [68]; the present work confirms this healing capacity of *Arnica m*. 2c (which corresponds approximately to the 4x used by those authors) also in macrophages, using a scratch-test model to evaluate cellular migratory events contributing to the *in vitro* wound healing process. This same model has previously been proven a valuable tool for assessing the effects of another homeopathic remedy, Calendula officinalis 3c, and of low-level laser therapy on human skin fibroblasts [69]. The increased mobility of the cells after treatment with *Arnica m*. can be due to many factors, including the augmented synthesis of chemotactic cytokines [22], and the ability to adhere to the surface of the well and to each other, also in virtue of the increased synthesis of ECM matrix.

At the present state of our knowledge, the mechanism of action of homeopathic medicines is extremely difficult to comprehend without the help of a suitable working hypothesis. On the basis of all the evidence available, the gene regulatory hypothesis originally proposed by Khuda-Bukhsh [70] offers an acceptable logical explanation of the molecular mechanism involved in the biological action of diluted homeopathic remedies in living organisms—whether plants or animals [71]. In experiments conducted in microbiological models ultradiluted *Arsenicum* 30c or *Arnica m*. 30c modified the expression of specific genes that are the targets of arsenite and UV irradiation injury, respectively [72–74]. Our studies [75,76] proved the extremely high sensitivity of the human neurocyte gene network to centesimal dilutions (2c, 3c, 4c, 5c, 9c and 30c) of *Gelsemium s*. Other experiments conducted on non-neoplastic epitelial prostate cell lines treated with Apis mellifica (honey bee) homepathic preparations reported modified expression of hundreds of genes after 24h incubation even with high dilutions 9c, 12c, 15c and 30c of the compound [77]. Genetic regulatory networks [78,79] may be the target of subtle messages by virtue of their flexibility in response to environmental stimuli. These findings support the hypothesis that homeopathic remedies could turn some important genes on or off, initiating a cascade of gene actions to correct the gene expression that has gone wrong and produced the disorder or disease. In this hypothesis the relevant target gene should be sensitive to similar stimuli and exert a pleiotropic transcriptional regulation on a battery of genes with related functions.

The slight effect in this *in vitro* model does not mean that the modulating effect will also be small *in vivo*, in whole organisms. Whereas conventional anti-inflammatory drugs are designed to suppress the underlying enzymatic mechanism of inflammation (e.g. prostaglandins, cytokines) and act at considerably high doses, homeopathic treatment is designed to regulate only the pathological aspects and malfunctioning tissues, because the inflammatory process in itself is seen as an expression of natural healing dynamics. In these conditions, even a 20–30% increase of macrophage activity in production of key-proteins such as fibronectin may have a decisive positive outcome of tissue healing and repair. Moreover, given the variety of *Arnica m*. effects and the multiplicity of its alkaloids, flavonoids, and sesquiterpene lactones [80], it is conceivable that the picture of its action is much more complex and could involve modulation of different cells and further pathways. The field of pharmacologic regulation of connective tissue and cell matrix by natural and chemical compounds is open to further studies and developments [46].

## Conclusions

The results of this work indicate that *Arnica m*. acts on macrophages by modulating a number of genes and by increasing cell motility. RNA-seq analysis allowed the identification of several genes which are particularly sensitive to ultra-low doses and high dilutions of this plant extract. Molecular analysis of gene expression suggests that a primary action of this medicinal plant is the stimulation of tissue matrix synthesis. These findings provide new insights into wound-associated molecular events and specifically point to macrophage fibronectin production as a potential therapeutic target of *Arnica m*. for the treatment of wound repair.

## Supporting Information

S1 Table Expression values (RPKM) of Control and *Arnica m*.-treated cells and differential expression (Log_2_ Fold Change) of the series of genes reported in Table 1. IL-4-differentiated THP-1 macrophages were treated with Control solvent or with *Arnica m*. 2c, 3c, 5c, 9c and 15c dilutions. Samples from Control solvent and *Arnica m*. 2c were analysed by RNA-seq in each experiment of five performed. RNA samples from 5 experiments of cells treated with *Arnica m*. dilutions 2c, 3c, 5c, 9c and 15 c were pooled, analysed with RNA-seq and Fold Change calculated comparing their RPKM with the mean RPKM of Control values.
(XLSX)

S2 Table Expression values (RPKM) and differential expression (Log2 Fold Change) of a series of extracellular matrix genes selected from the Reactome database as described in the text. The genes with FDR-adjusted p values > 0.05 and FDR unadjusted p values < 0.05 are here reported, while those with adjusted p values < 0.05 are reported in Table 1. Samples from Control solvent and *Arnica m*. 2c were analysed by RNA-seq in each experiment of five performed. RNA samples from 5 experiments of cells treated with *Arnica m*. dilutions 2c, 3c, 5c, 9c and 15 c were pooled, analysed with RNA-seq and Fold Change calculated comparing their RPKM with the mean RPKM of Control values.
(XLSX)
